# Construction and Application of Virtual Reality-Based Sports Rehabilitation Training Program

**DOI:** 10.1155/2022/4364360

**Published:** 2022-05-07

**Authors:** Huijun Yan

**Affiliations:** College of Sports, Henan Finance University, Zhengzhou, 450046 Henan, China

## Abstract

This paper adopts virtual reality technology to conduct in-depth research and analysis on sports rehabilitation training, designs a corresponding sports rehabilitation training program, and applies it to practice. An AR algorithm based on dynamic target tracking under VSLAM is proposed. The algorithm can effectively reject dynamic targets in static scenes while ensuring that the virtual objects registered based on dynamic template target tracking are still in the world coordinate system of VSLAM. To facilitate patients' hand function rehabilitation training, this paper uses OpenPose for 2D gesture pose recognition, combines camera pose information and depth information provided by VSLAM to map key points of the hand into the world coordinate system, and then completes the interaction by collision detection algorithm. The virtual interaction module is implemented in this paper to meet the demand for multiuser off-site interaction in virtual training. This paper uses the Unity3D software and Photon Server server to create a VR virtual scene and design a user interaction mechanism to realize a system that supports multiple users to train together online, which effectively extends the application scope of the VR training system. The module utilizes Unity3D's VR development capabilities to develop VR virtual basketball gym scenes and single-player offline interaction mechanisms such as virtual user single shooter and shooter; then, Photon Server is used to design and implement a multiuser remote login system and a multiuser interpass mechanism, thus achieving the effect of multiplayer remote online interaction in the same VR space. Finally, the proposed module was validated, and the results proved the effectiveness of the sports rehabilitation training program.

## 1. Introduction

After nearly a century of development, rehabilitation medicine has become an important part of the modern medical system “prevention, clinical treatment and rehabilitation” and a mature professional discipline, which refers to the integrated medical resources, using a variety of reasonable and effective means to help the injured, sick, and disabled to reduce and restore the physical and mental dysfunction caused by disease so that the patient can maximize the improvement and enhancement of mobility to return to the family and society [1]. This discipline is an integrated medical resource that uses a variety of reasonable and effective means to help reduce and restore the physical and mental dysfunction caused by the disease so that the patient's mobility can be improved and enhanced to the maximum extent possible and thus return to the family and society in the best condition. According to the World Health Organization (WHO), many disabilities caused by the disease are not predetermined or uncontrollable, and rehabilitation plays a key role in not only controlling or delaying the onset of disability but also speeding up the recovery process and reducing the negative consequences of many diseases. One of the external laser devices is made by making the tester wear a hair-triggerable headband and measuring the offset based on the laser light hitting the marked wall [2]. The results of the data measured in this manner are generally consistent with the cervical spine mobility reported in the medical literature for normal subjects. However, this approach requires keeping the patient at a certain distance from the marked wall, which has some inconvenience in terms of generating errors due to variations in vertical distance. Sensory abnormality is a general term for a group of mental disorders such as neurosis, obsessive-compulsive disorder, and anxiety disorders are all neurotic disorders. These symptoms usually have no pathological basis and are mainly psychiatric and psychological. Patients feel extreme pain, which can impede their psychological or social functioning. Some patients also experience symptoms of autonomic dysfunction, while others may present with dry, hyperkeratotic skin. On the other hand, the main method used in hospitals today is continuous X-ray photography, which allows the physician to view the characteristics of the cervical spine bones and the movement process by photographing the patient in a state of continuous motion. False-positive errors can also occur in impact diagnostics, and there are examples of cases where the imaging data from the X-ray film is not normal, but the test subject is not abnormal.

In addition to the application of VR technology in entertainment such as virtual laboratories, virtual nature sites, game entertainment, and movie production, close integration and good results have been developed in real industries such as military environment simulation and technical training, aircraft, and other vehicles driving training, medical surgery simulation, three-dimensional community planning, and geographic information systems. In recent years, with the development of VR technology, the demand for VR services in various industries is also increasing [3]. Thus, the realization of VR and its application system combined with other industries has important practical significance and economic value. During the development of modern society, the combination of sports and technology has gradually become one of the most active factors in the development of sports. Sports for all are becoming increasingly popular, and many sports types are gradually approaching the physiological limits of human beings, and the continuation of a large number of ineffective training makes more athletes suffer from injuries. The use of VR technology in virtual training has attracted considerable research attention. This can lead to the abandonment of sports training. Virtual technology, on the other hand, can be used to simulate real sports scenarios by computer, allowing athletes to train without fear of accidental damage and to understand the details of each technical movement through simulation, revising their movements for minor errors. The technology allows for more detailed breakdowns of difficult movements, with simulations allowing athletes to understand how to avoid damage when performing difficult movements. The results of virtual simulation training in sports such as soccer, sparring, Tai Chi, and Taekwondo have been widely used in world competitions. Various industries such as the military, firefighting, and sports are experimenting with developing virtual training systems to reduce training costs and increase their effectiveness.

Most patients with traumatic brain disease will have varying degrees of limb decline and motor abnormalities, mainly because their disease affects the normal cognitive function of the brain, and the common manifestations are mainly visual discrimination disorder, graphic discrimination difficulty, spatial relationship and spatial orientation disorder, motor perception disorder, etc. It is the damage to the cognitive level of the brain that directly leads to limb function limitation, motor impairment, and inability to take care of themselves. It is due to the cognitive impairment of the brain that patients have limited limb function, impaired movement, and inability to take care of themselves, and most of them also have cognitive impairments such as emotional, memory, and orientation. However, for various reasons, patients' motor cognitive rehabilitation care has received little attention in clinical treatment research, and the understanding of rehabilitation is generally characterized by traditional narrow-mindedness, i.e., only physical or limb function training and physical therapy are emphasized, while the importance of early psycho-cognitive treatment is ignored. The impairment of brain cognitive function affects the social adjustment ability of patients at the source and essentially hinders the comprehensive rehabilitation process of physical and psychomotor functions.

## 2. Related Works

Motor perception is one of the basic conditions for the survival of animals and humans, and it is biologically important. It helps individuals to recognize external environmental changes and receive biologically meaningful information through the perceptual system, thus helping organisms to establish the trajectory of external objects in the real world and to find their appropriate response methods. Therefore, motor perception is a basic cognitive ability that is necessary for human beings, both in daily life activities and in the process of performing motor skills [4]. Damage to motor neurons and motor perception affects patients' physical behavioral-motor abilities at the source [5]. In stroke patients, for example, more than 70% of patients with movement disorders have different categories of comprehensive cognitive impairment, which often directly affects the prognosis of patients' quality of life. The psycho-cognitive function has been proven to be plastic by medical research, and cognitive impairment can be sustained and effectively delayed and restored by human intervention and proper rehabilitation guidance [6]. Virtual reality technology is a computer advanced human-computer interface with immersion, interactivity, and conceptualisation as its basic features. It is based on computer technology and makes comprehensive use of computer 3D graphics technology, simulation technology, multisensor technology, multimedia technology, artificial intelligence technology, computer network technology, parallel processing technology, etc. It simulates the functions of human visual, auditory, tactile, and other sensory organs to produce an artificial virtual environment. In this virtual environment composed of computer graphics and multimedia technology, the user is able to interact with the computer system in real time through physical. In this virtual environment made up of computer graphics and multimedia technology, users can interact with the computer system in real time through physical, verbal, and other natural means, thus creating a multidimensional anthropomorphic information space, enabling people to immerse themselves in the virtual realm generated by the computer. Users can not only feel the “immersive” realism experienced in the objective physical world through virtual reality systems but can also break through the constraints of space, time, and other objective conditions and feel experiences that cannot be experienced in the real world.

The movements of Tai Chi experts are captured, and the captured movements are delivered to students in a multimodal format in immersive rooms, HMDs, and regular PC environments. Students' movements are also captured for quality assessment and are used to form a virtual collaborative learning atmosphere. In addition to this, a virtual reality ski training system using an indoor ski simulator is proposed. The system is based on a simple indoor ski simulator with two trackers to capture the motion of the skis [7]. Through simulation technology, the teaching experimental equipment, instruments, and environment in the real environment are restored 1 : 1 to the virtual world, categorized and designed with certain logical rules according to the links and processes of experimental teaching, and a virtualized and shareable experimental teaching scenario is constructed with the help of interactive means and network technology [8]. This algorithm uses error diffusion to achieve dithering by scanning the pixels of the image from left to right and top to bottom and normalizing (or binarizing) them one by one, superimposing the errors resulting from the normalization of the pixels onto neighbouring pixels, without affecting the pixels that have already been processed. The effect of this is that if some pixels are rounded down, it is more likely that the next pixel will be rounded up, thus minimising the average quantization error. In addition, the teaching form of virtual simulation experiment can also get rid of the restrictions in time, space, and resources, so as to meet the diversified needs of experimental teaching users and can train their skills by replaying professional skiers [9]. The training system consists of three modules: a trainer replay system to review the movements of the professional skier, a time control system to watch the detailed movements of the trainer and the user, and a visualization module to compare the differences in movements between the user and the trainer [10].

In a virtual exercise experiment comparing the training benefits of virtual exercise from different perspectives, this study found that the more immersive first-view training significantly enhanced trainers' motivation and riding speed [11]. The experiment used virtual opponents for virtual obstacle running training, and virtual training was found to improve trainers' decision-making ability and enhance athletic performance by rating speed, stride count, and decision-making ability [12]. Believing that competitors in a virtual environment can directly induce stress during exercise and thus improve athletic performance, his team also compared the different athletic performances of older adults during virtual cycling training alone and when competing with a virtual opponent, who was asked to try to outperform the virtual opponent, and their findings showed that the trainer's cycling output power was higher when competing with a virtual opponent than when cycling alone. The virtual reality walking smart training table was first used in the training of healthy elderly people to improve their balance and reduce the risk of falls, and in recent years, it has been gradually used in the training of stroke patients and amputee patients. The training concept of C-MILL VR+ comes from the theory of motor control and learning, and its advantages are accurate recording of the user's spatio-temporal parameters of each step and showing them to the user and the operator in various forms; real-time display of dynamic data to the operator; support for real-time projection-guided adjustment, assessment of posture control, and training to lay the foundation for gait; and its basis task-oriented design, emphasizing the inclusion of feedback mechanisms in each game, taking into account the cognitive and somatic levels of training games.

## 3. Analysis of the Application of Virtual Reality for the Construction of Sports Rehabilitation Training Programs

### 3.1. Virtual Reality Technology for Sports Rehabilitation Training

The basic components of a VR device are divided into two basic modules: the computation module, the display module, and the precision positioning module, which are used to render and output images; the display module, which generally consists of two screens placed on the left and right eyes, electronic optical components (magnifying glass and diopter myopia) and gyroscopes, is used to display. The calculation module calculates and transmits the image and provides the head action position; the precise positioning module generally consists of VR handle, head-mounted display, and base station, the VR handle provides the hand action position, the head-mounted display provides the head action position, and the base station provides the auxiliary positioning role, together to complete the positioning function. The alignment method first converts the depth plane coordinates to depth camera space coordinates using the depth camera internal reference matrix, then converts the depth camera space coordinates to RGB camera space coordinates using the external reference to calculate the rotation and translation matrices, and finally converts the RGB camera space coordinates to RGB plane coordinates using the RGB camera internal reference matrix.

The inside-out tracking technology, which does not require the installation of additional locators, relies only on the plural cameras on the headset to complete the positioning function [13]. The principle relies on optical tracking, through the installed plural cameras, allowing the device to detect changes in the external environment and calculate the spatial location of the cameras through a vision algorithm. Taking two cameras as an example, the mode in which two cameras are positioned is called binocular mode, named because it works like two human eyes. As shown in Figure 1, the parallax *d* is defined as the difference between the horizontal coordinates of the pixels of point *M* in the left and right images, and the *Z*-axis coordinates of point *M* in the figure can be derived using these two similar triangles, which is the depth value.

By alternating the horizontal-vertical laser between the base stations, the angles of these sensor points in the coordinate system of the base station can be calculated based on the time of flight if the horizontal-vertical laser beam is swept over enough sensor points in one cycle, and thus, the coordinates of the laser-irradiated sensor points in the projection plane can be obtained. Also, considering that the laser-scannable points on the sensor are known concerning the orientation of the sensor, it is possible to calculate the rotation and translation of the laser-scannable sensor point phase in the base station coordinate system and thus obtain the coordinates of the points on the sensor. Together with the attitude obtained on the Inertial Measurement Unit (IMU), the attitude and position of the illuminated sensor point can be given more accurately. The Inertial Measurement Unit, which combines various sensors with gyroscopes, is used to detect the rotation and motion of the three axes.

Depth image and color image alignment are an essential prerequisite in the calculation of the standard angle of human cervical spine activity. We can only get the image coordinate system position of the pixel where the feature point is in the color image, not necessarily the corresponding depth data, and only after the depth image and the color image are aligned is it meaningful to process the color image. There are two types of alignment between depth image and color image according to different benchmarks; one is based on color image, and the other is based on the depth image. To avoid the lack of feature points in the color image after alignment, this paper uses the alignment method based on the color image. Therefore, in this paper, we first align the depth image and the color image with the color image as the reference. Under normal use, the host computer software will directly open COM3 for communication. In order to realize the listening function, the virtual serial port pair and the listening software are added. Instead of connecting directly to the physical serial port, the host computer connects to one end of the virtual serial port and uses the listening software to open the physical serial port and the other end of the virtual serial port to realize the data transmission and listening function. The depth data of the color image feature points are obtained from the aligned depth image, and the two-dimensional point set can be converted into a three-dimensional point set, and the coordinate system is a three-dimensional spatial coordinate system with the depth camera as the origin.

The principle of aligning two images is to first convert the points in the depth image to three-dimensional coordinates and then project the three-dimensional coordinates onto the color image. The pixel coordinate system of an image conventionally takes the upper left corner of the image as the origin, and the pixel coordinates are generally expressed in *u*, *v*. The origin of the camera coordinate system is the camera optical center, and it is known from the imaging principle that assuming that the object *P* has coordinates [*x*_*c*_, *y*_*c*_, *z*_*c*_]^*T*^ in the camera coordinate system, the object is in the image coordinates *Pu*, *v*[*u*, *v*]^*T*^ as *u* = *f*(*x*) − *xz* + *Cx*, *v* = *f*(*y*) − *xz* + *Cx*, *f*(*y*) are the camera focal lengths, and [C*x*, *Cy*]^*T*^ is the translation of the origin of the camera coordinate system to the origin of the pixel coordinate system, expressed in matrix form as follows:

(1) $$\begin{array}{c} \left[\begin{array}{c} u\\ v\\ 1 \end{array}\right]=\frac{1}{z}\left[\begin{array}{ccc} fx & 0 & Cx\\ 0 & fy & Cy\\ 0 & 0 & 1 \end{array}\right]\left[\begin{array}{c} xc\\ yc\\ zc \end{array}\right], \end{array}$$

where the matrix *K* is called the internal parameter matrix of the camera. Let the position of the object in the camera coordinate system be

(2) $$\begin{array}{c} \left[\begin{array}{c} xc\\ yc\\ zc \end{array}\right], \end{array}$$

in the world coordinate system, since the camera also has the position and pose, the world coordinates of the object (denoted as Pw) need to be transformed according to the current pose of the camera, expressed by the rotation matrix *R* and the translation vector *t*. The transformation relation is

(3) $$\begin{array}{c} P_{u,v}=\left[\begin{array}{c} u\\ v\\ 1 \end{array}\right], \end{array}$$

(4) $$\begin{array}{c} P_{c}={RP}_{w}^{2}-t. \end{array}$$

The skeleton data collected by Kinect sensors belong to the camera coordinate systems of different Kinect sensors. To facilitate the unification and fusion of skeleton data collected by different Kinect sensors, their coordinate systems need to be unified [14]. Therefore, the rotation matrix and displacement vector of each Kinect sensor must first be obtained by calibration to convert them to the global coordinate system for unification to integrate the skeleton data. Some work has chosen to unify the coordinate systems of different Kinect cameras into one of the Kinect coordinate systems, which has the advantage of facilitating the computation but not the presentation of the final skeletal data in a variety of different views. The advantage of fusion from the global coordinate system is that the skeletal data can be more easily converted to various viewpoints.

In the process of motion capture and recognition, users with different body sizes are encountered. The position of each skeleton point acquired by Kinect is based on the user's body size, so even if two different users do the same action, the final recognition result may be misclassified due to the change in body size. Therefore, in this section, the joint position data of the fused skeleton is normalized so that it remains constant with the size of the trainee's body. In this section, 24a limb is defined and described, and an ergonomic kinematic tree consisting of 25a joint and 24 a limb is considered. The joints and limbs are described by nodes and edges, respectively, and the “SpineBase” node (*j* = 1) is used as the root node of the kinematic tree.

(5) $$\begin{array}{c} w\left(s_{j,f}\right)=\left\{\begin{array}{c} 1.0,s_{j,f}isnkone\\ 2.0,s_{j,f}iskone\\ 3.0,s_{j,f}isnone \end{array}\right.. \end{array}$$

In this paper, we obtain the final fused skeletal data by considering the error and the tracking quality of the Kinect camera with a weighted fusion method.

(6) $$\begin{array}{c} P=\frac{\sum_{f\in F}w\left(s_{j,f}\right)\mu \left(d_{j,f}\right)}{\sum_{f\in F}w\left(s_{f,f}\right)\mu \left(d_{f,f}\right)}. \end{array}$$

In this paper, we use the positioning module in HTC Vive to obtain the motion data of the subject's neck by putting the subject on the HTC Vive head-mounted display device and using the positioning module to position the head in real-time. In this paper, we use the Unity software to obtain the real-time positioning data of the VR device, and we use three groups of movements: cervical flexion and extension, left and right tilt, and left and right rotation, to obtain the initial angular difference of the subject's cervical mobility. Unity generally uses quaternions (Unity's Rotation property), which are complex numbers used to represent rotations in 3D space, to record the pose of VR devices. A quaternion *q* has one real and three imaginary parts and is represented as follows.

(7) $$\begin{array}{c} q=q_{r}-q_{i}i+q_{i}j-q_{i}k. \end{array}$$

For the measurement of cervical spine activity, the key is the angular change between the postures returned by the two head-mounted displays, which is the angular difference between the two quaternions. To calculate the angular difference between the two quaternions *q*_1_, *q*_2_, the difference between the quaternions qd is calculated using Equation (8) and then reduced to a readable angle as follows:

(8) θ=arccotqii2+qji2−qki2qr.

The server-side uses the same development language and libraries as the client-side and is mainly responsible for receiving data from the client-side Kinect, initializing, and calibrating multiview data, and fusing data, so the main functions of the server-side can be divided into data reception and reading module, a data calibration module, and data fusion module [15]. The relationship between the three modules on the server side is shown in Figure 2. In the initialization phase, the server detects whether the Kinect is connected to each viewpoint and whether there is a target in the respective viewpoint.

The data reception module receives data from each client, and when no target is detected in the data from all clients, the server continues to listen in the data reception module until at least one client detects the target. If the target is detected to have moved during the process, the module will be recalibrated; if the target is not detected after the module is completed, it will be returned to the data receiving module for listening. After the data calibration is completed, the converted data is fused in the data fusion module and displayed.

The client data is transmitted via TCP/IP protocol and received on the server-side in the form of “Kinect Serializer” serialization. Since this module and the data transmission function of the client function is in a send/receive relationship, the initialization and connection establishment process of both is the same, and the main difference between the data reception module and the data transmission function of the client function is the core code of the reception part.

First, the user performs the test pose in the motion capture system separately, and the client and server record the skeleton information from their respective viewpoints. Firstly, when the user faces the A-camera, the head of the user is deviated from the A-camera view due to the position of the user and the tracking error of Kinect, and the legs are not well tracked due to the distance problem but can still be observed; the skeleton obtained by the multiview motion capture system proposed in this paper corrects the head deviation from the A-camera view and improves the tracking effect of the legs.

### 3.2. Application Design of Physical Rehabilitation Training Program Construction

Rehabilitation treatment is a long, staged, complex movement process in which multiple approaches are involved and can constitute an experiential stage of beginning, development, and completion concerning the temporal dimension, in line with the three experiential dimensions of expectation, process, and impact in the EEI model of experiential design. Rehabilitation therapy technology is a new therapeutic discipline that promotes the physical and psychological rehabilitation of injured patients and people with disabilities, as well as a new technical specialism. Its aim is to enable people to regain as much as possible their ability to perform their daily activities, study, work, and labour, as well as their social life, to integrate into society and to improve their quality of life. The rehabilitation movement expectation is the beginning of the whole rehabilitation experience in which the patient is psychologically prepared to accept or stimulate the rehabilitation event, which includes the patient's inner desire to meet the rehabilitation needs, behavioral motivation and goals, behavioral intention, encouragement, persuasion from family and friends, and reputation of hospital evaluation [16]. It is the main part of the rehabilitation movement, which involves the interaction process of people in the whole rehabilitation situation, and the objects of interaction include rehabilitation products, rehabilitation services, rehabilitation space, and the clinicians, rehabilitation therapists, patients' families, administrators, government, and other related stakeholders. The rehabilitation movement impact refers firstly to the recovery and improvement of the patient's motor perception and the closely related physical movement ability to a certain extent, and secondly, and more importantly, to the cognitive results and emotional continuity obtained by the patient's reflection on the event after discharge from the hospital, and the rehabilitation experience can be concluded when it is settled into a unique memory and developed into a unique story belonging to the patient. Physical rehabilitation training is a training activity in which the user transmits his/her movements into the computer through input devices (e.g., data gloves and motion capture devices) and receives visual, auditory, or tactile feedback from the output feedback devices to ultimately achieve maximum recovery of some or all of the patient's body functions. This training method not only greatly saves human and material resources for training but also effectively increases the fun of treatment, stimulates the patient's enthusiasm to participate in treatment, changes passive treatment into active treatment, and improves the efficiency of treatment.

In the process of rehabilitation experience, whether with others, with the product, or with the whole space, patients need to transmit information to each other in the process of interaction, which can be in various forms of transmission such as expression, words, graphics, color, or form changes. The feedback from patients can be a smile or a word of encouragement from the doctor; with products, it can be a flashing light or a prompt from the interface; with space, it can be a prompt of spatial information, a change of light, a change of path, etc. Different feedback forms are needed in different contexts. Only when the patient gets the feedback can he or she have a certain grasp of the situation of his or her current operation and can also start planning the next operation, which helps the patient to complete the task and reach the goal [17]. The patient's expectation of getting feedback also varies according to the patient's characteristics, difficulty, and frequency of use. For example, if the patient performs arm exercise training every day, he does not expect to get encouragement from others every time he completes it; instead, for him to complete a competitive competition with others, he psychologically strengthens his expectation of feedback. Patients were originally due to illness and mood fluctuations, so in the design process, the designer should fully consider the factors in the interaction, including the object of feedback, frequency, and form, to promote the positive interaction between the patient and the environment, which helps the patient's emotional control, as shown in Figure 3.

Subjects were seated with their heads in a neutral position, and the cervical spine range was measured using an orthopedic goniometer. During the acquisition, vertical and horizontal lines were marked on the walls and floor (this experiment utilized vertical and horizontal lines already present in the hospital setting) to serve as a reference for neck motion and orthopedic goniometer placement. The axis of the orthopedic goniometer was first placed along the sagittal plane at the top of the mastoid process to test the neck flexion angle and extension angle. Then, the range of lateral tilt of the neck to the left and right was measured using the orthopedic goniometer axis located on the spinous process of the seventh cervical vertebra. A final check of the neck rotation to the left or right is performed with the axis of the orthopedic goniometer located in the center of the head. The measurement of the subject using the orthopedic goniometer needs to be performed twice, using the maximum value for recording. Decreased muscle strength is a reduction or loss of casual motor function and refers to a decrease in the strength, amplitude, and speed of muscles during active movement. The different degrees of muscle weakness can be divided into complete paralysis and incomplete paralysis (i.e., light paralysis). Monoparesis is most often seen in poliomyelitis; hemiparesis is often accompanied by damage to one side of the cranial nerve, most often due to intracranial damage or stroke; crossed hemiparesis is paralysis of one limb and damage to the opposite cranial nerve, most often due to brainstem lesions; paraplegia is transverse spinal cord injury, most often due to spinal cord trauma and inflammation. In addition, the intra- and intergroup agreement of the orthopedic goniometer was not examined in this study because the consistency of the cervical mobility measured by the orthopedic goniometer has been well established in previous studies.

The computer generates white rectangles and red-white rectangles based on the gait parameters detected during the warm-up phase, the size of which is determined by the subject's foot length, projects them onto the treadmill via a projector and forms stepping targets (white rectangles) and ducking targets (red-white rectangles) as ducking targets, and the computer provides the patient with rhythmic auditory cues matching the speed during the walk. The computer gives the patient a rhythmic auditory cue that matches the speed and a red-green visual cue that matches the success of stepping or dodging. The patient is asked to step on and avoid the target as accurately and rhythmically as possible during the walk.

The computer-generated different color square highlighting area and projected on the treadmill, according to the patient's condition, selectively sets and adjusts the time and frequency of the square appearing. If the patient is not in the square area, the system gives a sound to remind him/her to adjust the speed as soon as possible to ensure that he/she is in the area, as shown in Figure 4.

The outermost contour of the hand is identified after binarization of the hand, and the convex packets corresponding to the set of hand contour points are detected and drawn. For a convex wrap curve, the curve is always convex, or at least flat [18]. If there is a concave part, it is called a convex defect. The hand convex defect area is the gap area formed between the convex wrap curve and the hand contour line. The intrinsic function detects the hand convex defect and obtains the return array including the starting point, the endpoint, the deepest point (i.e., the point with the largest distance from the hand contour point to the convex wrap curve in the same defect area), and the approximate distance from the convex wrap curve to the deepest point for each defect area.

The rehabilitation motor impact layer is a transformation of the patient's motor ability, lifestyle, or life trajectory after treatment, and the experiential impact is characterized by long-term uncertainty. From the individual level of rehabilitation, the rehabilitation experience was no longer a forced and painful treatment experience, but another form of participation in social interaction, where they are treated while the need for environmental adaptation becomes friendly and adjustable so that the patient's movement is not limited by the disease; from the social level of rehabilitation, paying practical attention to the patient's wishes and needs and balancing the demands of relevant stakeholders under the rehabilitation public space are social. In terms of the social aspect of rehabilitation, it is necessary for the long-term development and progress of rehabilitation medicine.

## 4. Analysis of Results

### 4.1. Performance Design of Virtual Reality System for Physical Rehabilitation Training

In this paper, the person who recorded measurements on the depth camera-VR device and the orthopedic protractor is referred to as the observer, and the person who performed the measurements using the hybrid device, as well as the orthopedic protractor, is referred to as the subject. The difference obtained from the results of two tests performed by the same observer on all subjects using the hybrid measurement of the depth camera-VR device is called the intragroup variation of that measurement and is expressed as the intragroup mean variation. The difference in measurement results obtained by different observers using the same measurement method on the same subject is the interobserver variation and is expressed as the average between-group variation.

Intragroup reliability of the depth camera-VR device hybrid measurement data was calculated from the first and second measurements of all subjects using the depth camera-VR device, while interobserver reliability was assessed based on the first measurement out of two observers for each subject. Data were analyzed by a two-way random model and expressed by the intragroup correlation coefficient (I ICC) using a two-way random-effects model and its 95% confidence interval (CI). The standard error of measurement was calculated using the following formula: the square root of the difference between the ICC and 1 multiplied by the standard deviation derived from the two measurements, as shown in Figure 5.

The plot can also be used to investigate the variability and correlation between the measured values of the two measurement methods to detect potential systematic bias and identify outliers. *x* and *y* axes represent the mean of the measured values of the corresponding measurement methods and the difference between their measurement method data, respectively. Limits of Agreement (LoA) are defined as the mean difference ± 1.96 standard deviation. The Coefficient of Repeatability (COR) is equal to 1.96 standard deviations of the difference between the data obtained by the two measurement methods and is used to represent the difference in measurement accuracy with the orthopedic goniometer and the depth camera-VR hybrid device. A paired *t*-test was performed to compare the mean difference between the two assessments, a Pearson correlation analysis was also performed on the data obtained by the two methods, and a *p* value < 0.05 was considered significant. The general group used conventional care, such as detailed examination of the patient's physical signs. The observation group used early rehabilitation nursing interventions, with the following care measures: firstly, psychological support. The prevalence of stroke disease is usually very acute, with prominent clinical manifestations, and many patients also experience more significant language and physical impairment after the disease, making the patient more agitated and negative emotions occur.

In this paper, we analyze the mean intragroup variance and mean intergroup variance of the mixed measurement data of the depth camera-VR device, analyze the interobserver variance of the mixed measurement modality, and finally analyze the difference between the results of the mixed measurement modality and the orthopedic protractor measurement modality, as shown in Figure 6.

The consistency of the mixed depth camera-VR device measurement approach was better for the same observer for the same subject in both measurements, with significant differences in the reliability of the subject's scores in the supination, flexion, and right rotation directions for two different observers. The mean difference was 1.885, *p* = 0.040 in the supination-extension direction, 1.681, *p* = 0.047 in the flexion direction, and 2.410, *p* = 0.006 in the right rotation direction. The reasons for the significant differences were speculated to be, firstly, objective differences in the actual cervical mobility of the different measurers; secondly, from the measurement method, different measurers may have the measurement process; there may be head and neck fatigue, which is caused by different levels of fatigue in each individual; there are also subtle changes in the range of motion during the measurement process as the subjects completed the warm-up during the previous measurement.

However, it can be seen from the graph that these differences are largely negligible, and the accuracy of the present measurement is high. The 6 ICC for the same subject ranges from 0.894 (9595% CI, 0.801 to 0.945) in the left lateral tilt direction to 0.954 to 0.988 in 0.977 the supination direction and from 0.39 to 1.045 and 1.081 to 2.896 in the SEM and MDC; the ICC ranges between 0.676 (95% CI, 0.446 to 0.822) and 0.909 (% CI, 0.827 to 0.953) in the measurements of two different subjects. The reliability of the method in this paper is good in terms of repeatability measurements, and its consistency is also good.

It has showed that only 2 of the 35 subjects in supination and extension, 2 in flexion, 2 in left rotation, 1 in right rotation, and 2 in left lateral tilt exceeded the 95% confidence interval. These data demonstrate the consistency of the two measurements in the different directions of cervical spine motion. The repeatability coefficients for cervical spine motion in different directions ranged from 6.628 to 9.527. Regarding where there are some outliers between the VR device and the protractor, probably due to measurement differences, the results are acceptable overall. Rehabilitation is a process that requires interaction with the environment in movement and restoration of behavioral capacity. The aim is to create a dynamic, active, and continuous state of rehabilitation that promotes continuous satisfaction and growth in the patient's interaction with the environment, resulting in an enjoyable rehabilitation experience. Movement is the basic form of existence of all things, and kinesthetic perception is a basic cognitive ability of human beings to recognize and identify movement information and to respond to it accordingly.

### 4.2. Results of the Rehabilitation Training Program Application

Measuring cervical spine motion is more challenging than assessing peripheral joint motion. Cervical spine motion is three-dimensional and is not limited to a single plane. Motion in one axis may be influenced by other dimensions. In addition, cervical motion involves multiple joints; therefore, the estimated range of cervical spine mobility may change significantly when the reference joints are different. After the experiments in this paper, it was found that the measurement method used in this paper can reliably measure cervical spine mobility in six directions, with ICC ranging from 0.894 to 0.977 within groups and from 0.676 to 0.909 between groups. It is hypothesized that the satisfactory results are not only due to the use of a depth camera-virtual device mix for measurement data but also attributed to the availability of relatively standardized subject homogeneity data. Although there were some significant interobserver differences in the supination, flexion, and right rotation directions, the average differences were small. The SEMs for all six directions of neck motion measured using the depth camera-VR device mix were within 1.045°, indicating the high measurement accuracy of this measurement method, as shown in Figure 7.

Regarding the agreement between the measurements and the orthopedic goniometer in this paper, the Bland-Altman plot shows excellent agreement, with at most two out of 35 paired measurements in the 95% confidence interval not falling within the confidence interval. However, for neck flexion, pinpointing the center of the head may be difficult. In addition, the angle of head rotation depends on the vertical axis of the occipito-axial joint. Therefore, rotational head motion in the horizontal plane may not be measured accurately if measured with an orthopedic protractor. However, these factors are unlikely to affect the measurements used in this paper because the VR device uses an indoor positioning system and IMU device fusion to estimate the position of the target in 3D space.

There was no statistically significant difference between the test group and the control group in terms of 1010 meter walking speed (10 mWT) before treatment (*p* > 0.05); intragroup comparison between the test group and the control group showed a highly significant difference (*p* < 0.01), indicating that the meter walking speed (10 mWT) in both groups improved significantly after weeks of treatment. Suggesting that the test group improved the meter walking speed more significantly than the control group, as shown in Figure 8.

This trial proved that the virtual reality intelligent running table training program and conventional exercise therapy have positive effects in improving the lower limb motor function, balance function, and walking ability of stroke patients, but the rehabilitation efficacy of virtual reality intelligent running table training is better than conventional exercise therapy training, and the positive role of virtual reality intelligent running table in the rehabilitation of stroke patients is determined. It is a new and effective treatment method for stroke patients, which has practical application value and clinical significance, as well as saving medical resources and social costs, and has social significance.

## 5. Conclusion

In this paper, an interactive limb training system is designed for the functional characteristics and training requirements of a mobile rehabilitation training robot, which mainly includes a mechanical training module for the lower limbs, a virtual interactive training module for the lower limbs, and a virtual interactive training module for hand grasping. For the rehabilitation of the lower limbs, the system is suitable for all stages of rehabilitation training, but for the rehabilitation of the hand, it is more suitable in the later stage of rehabilitation, i.e., the patient can train the finger joint movement ability of the hand independently at this time, so that it can better approach the normal level. The design strategy of the product experience focuses on establishing the patient's active, correct, and self-regulated movement pattern; the service strategy emphasizes the patient's pleasant and autonomous movement state and the guidance of the dynamic balance of spatial relationships, encouraging the individual to actively participate in the collective and society; the spatial environment strategy places more emphasis on the overall movement perception and the continuous and smooth kinesthetic experience of space. Adhering to such logic and principles, specificity design strategies for different experience levels are proposed, respectively. In the simulation environment displayed by virtual reality technology, different training scenarios are provided for patients who need to cross obstacles and complete the S-shaped path, and the length and width of obstacles that need to be stepped over can be set according to different conditions of patients, thus promoting the improvement of stride length, step speed, step width, and step frequency. Applying the virtual reality exercise tablet training system to the patient, the patient walked on the exercise tablet while avoiding virtual obstacles, and through 5 weeks of training, the patient's 2 min stride test improved by 9.5%, and the quadratic stride test improved by 13%.

## Figures and Tables

**Figure 1:** Principle of binocular model.

**Figure 2:** Relationship between server modules.

**Figure 3:** Initial angular difference in cervical spine mobility of the subjects.

**Figure 4:** Change of hand contour surface hedge in vertical position.

**Figure 5:** Speed time diagram of the second experiment of cervical spine angle measurement with the hybrid depth camera-VR device.

**Figure 6:** Intra- and intergroup evaluations and corresponding differences in cervical spine mobility measured with the depth camera-VR device hybrid.

**Figure 7:** Bland-Altman diagram of cervical mobility measured by orthopedic goniometer.

**Figure 8:** Comparison of two groups of 10 mWT.

## Data Availability

The data used to support the findings of this study are available from the corresponding author upon request.

## References

[1] An M. Y., Ko K. A., Kang E. J. (2020). Problems and directions of development through analysis of virtual reality-based education in Korea. *International Journal of Information and Education Technology*.

[2] Ryu J. J., Kang S. J. (2021). Virtual reality based fall training system. *Journal of the Korea Institute of Information and Communication Engineering*.

[3] Yang Y. (2018). The innovation of college physical training based on computer virtual reality technology. *Journal of Discrete Mathematical Sciences and Cryptography*.

[4] Checa D., Bustillo A. (2020). A review of immersive virtual reality serious games to enhance learning and training. *Multimedia Tools and Applications*.

[5] Pourazar M., Bagherzadeh F., Mirakhori F. (2021). Virtual reality training improves dynamic balance in children with cerebral palsy. *International Journal of Developmental Disabilities*.

[6] Sattar M., Palaniappan S., Lokman A., Shah N., Khalid U., Hasan R. (2020). Motivating medical students using virtual reality based education. *International Journal of Emerging Technologies in Learning (iJET)*.

[7] Mihajlovic Z., Popovic S., Brkic K., Cosic K. (2018). A system for head-neck rehabilitation exercises based on serious gaming and virtual reality. *Multimedia Tools and Applications*.

[8] Mbada C. E., Makinde M. O., Odole A. C. (2019). Comparative effects of clinic- and virtual reality-based McKenzie extension therapy in chronic non-specific low-back pain. *Human Movement*.

[9] Felipe L., Hunnicutt S. (2020). Virtual reality as a vestibular rehabilitation tool for athletes after concussion: a literature review. *Advances in Rehabilitation*.

[10] Vibhuti V., Kumar N. (2021). Realisation of a virtual reality based remedial module for cognition and hand function rehabilitation. *Journal of Scientific and Industrial Research (JSIR)*.

[11] Köyağasıoğlu O., Özgürbüz C., Bediz C. Ş., Güdücü Ç., Aydınoğlu R., Akşit T. (2022). The effects of virtual reality nonphysical mental training on balance skills and functional near-infrared spectroscopy activity in healthy adults. *Journal of Sport Rehabilitation*.

[12] Juras G., Brachman A., Michalska J. (2019). Standards of virtual reality application in balance training programs in clinical practice: a systematic review. *Games for Health Journal*.

[13] Burcal C. J., Haggerty A., Grooms D. R. (2021). Using virtual reality to treat perceptual and neurocognitive impairments after lower extremity injury. *Athletic Training & Sports Health Care*.

[14] Wang H., Wu J. (2021). A virtual reality based surgical skills training simulator for catheter ablation with real-time and robust interaction. *Virtual Reality & Intelligent Hardware*.

[15] Pourazar M., Mirakhori F., Hemayattalab R., Bagherzadeh F. (2018). Use of virtual reality intervention to improve reaction time in children with cerebral palsy: a randomized controlled trial. *Developmental Neurorehabilitation*.

[16] Lina C., Guoen C., Huidan W. (2020). The effect of virtual reality on the ability to perform activities of daily living, balance during gait, and motor function in Parkinson disease patients. *American Journal of Physical Medicine & Rehabilitation*.

[17] Moon K. J., Han K. H. (2018). Review on the articles of the effect of image training program with 3D virtual reality and use for physical activity of older adults: based on the embodied cognition. *Journal of the Korean Applied Science and Technology*.

[18] Kakavas G., Malliaropoulos N., Bikos G. (2021). Periodization in anterior cruciate ligament rehabilitation: a novel framework. *Medical Principles and Practice*.

